# A Chinese herbal formula, Jian-Pi-Yi-Shen decoction, improves muscle atrophy via regulating mitochondrial quality control process in 5/6 nephrectomised rats

**DOI:** 10.1038/s41598-017-10027-4

**Published:** 2017-08-23

**Authors:** Dongtao Wang, Jianping Chen, Xinhui Liu, Ping Zheng, Gaofeng Song, Tiegang Yi, Shunmin Li

**Affiliations:** 1 Department of Nephrology, Shenzhen Traditional Chinese Medicine Hospital, Guangzhou University of Chinese Medicine, Shenzhen, 518033 China; 2 Shenzhen Key Laboratory of Hospital Chinese Medicine Preparation, Shenzhen Traditional Chinese Medicine Hospital, Guangzhou University of Chinese Medicine, Shenzhen, 518033 China; 3 Department of Nephrology, Ruikang Affiliated Hospital, Guangxi University of Chinese Medicine, Nanning, 530011 China

## Abstract

Muscle atrophy is one of the serious complications of chronic kidney disease (CKD). Dysregulation of mitochondrial quality control (MQC) process, including decrease mitochondrial biogenesis, impair mitochondrial dynamics and induce activation of mitophagy, play an important role in mediating muscle wasting. This study aimed to observe effects of Jian-Pi-Yi-Shen (JPYS) decoction on muscle atrophy in CKD rats and explore its possible mechanism on regulation of MQC processes. The 5/6 nephrectomised rats were randomly allocated into 2 groups: CKD group and JPYS group. Besides, a sham-operated rats as sham group. All rats were treated for 6 weeks. Results showed that administration of JPYS decoction prevented body weight loss, muscle loss, muscle fiber size decrease, muscle protein degradation, and increased muscle protein systhesis. In addition, JPYS decoction increased the mitochondrial content and biogenesis proteins, and down-regulated the autophagy and mitophagy proteins. Furthermore, JPYS decoction increased mitochondrial fusion proteins, while decreased mitochondrial fission proteins. In conclusion, JPYS decoction increased mitochondrial content and biogenesis, restore the balance between fission and fusion, and inhibited autophagy-lysosome pathway (mitophagy). Collectively, our data showed that JPYS decoction to be beneficial to muscle atrophy in CKD, which might be associated with the modulation of MQC process.

## Introduction

Chronic kidney disease (CKD) is characterized by a progressive loss in renal function over a period of months or years. Enormous studies have been demonstrated that its action mechanism is related to the excessive accumulation of extracellular matrix and podocyte loss and inflammation as well as the dysfunctions of lipid metabolism and amino metabolism^1–6^. A few reports indicated that CKD is associated with muscle atrophy, which directly correlates with mortality and morbidity^7^. Potential stimuli of muscle atrophy in CKD include acidosis, angiotensin II production, inflammation, up-regulation of the ubiquitin-proteasome and autophagy–lysosome systems (UPS and ALS), and dysregulation of mitochondrial quality control (MQC) processes^8, 9^. Unfortunately, preventive and therapeutic interventions that block muscle atrophy are still at the initial stages of development. More and more patients accepted complementary or alternative therapies such as traditional Chinese medicine (TCM)^10–14^. We examined whether a traditional Chinese medicine, Jian-Pi-Yi-Shen (JPYS) decoction, would prevent muscle atrophy by modulating the MQC process.

The UPS is recognized as the major contributor to muscle proteolysis, responsible for 50% or more of total protein degradation in skeletal muscle. The UPS is the major intracellular protein degradation pathway, which can degrade the myofibril proteins into its components (actin, myosin, troponin, and tropomyosin)^15^. These proteins are targeted and degraded by two muscle-specific E3 ubiquitin(Ub) ligases, muscle atrophy F-Box (MAFbx/Atrogin-1) and muscle-specific RING finger protein (MuRF1)^16, 17^. Parallel to the above pathway, the ALS is believed to target and cleave long-lived proteins, bulk cytoplasm and organelles through the lysosomal machinery^18^. The activation of UPS and ALS-related genes is normally blocked by Akt through negative regulation of Forkhead box O (FoxO) transcription factors, including FoxO1, FoxO3a and FoxO4. The translocation and transcriptional activity of FoxO members is sufficient to increase atrogin-1 and MuRF1 expression, and cause muscle atrophy^19^.

MQC processes are tightly regulated by several processes, e.g. biogenesis, fusion, fission, and mitophagy. It is reported that chronic diseases activate a mitochondrial response that ameliorate the “quality” of skeletal muscle mitochondria cells at different molecular levels: (i) biogenesis through the action of the key regulators peroxisome proliferator-activated receptor gamma coactivator 1-alpha (PGC-1α), nuclear respiratory factor 1/2 (NRF-1/2), adenosine 5′-monophosphate (AMP)-activated protein kinase (AMPKα), and ATP synthesis; (ii) dynamics by the mitochondrial remodeling GTPase proteins such as mitofusin-2 (Mfn-2) and optic atrophy 1 (OPA-1) for fusion and dynamin-related protein 1 (DRP-1) and fission 1 (Fis-1) for fission; (iii) turnover of damaged mitochondria by mitophagy through PTEN induced putative kinase 1(PINK1), Parkin and Bnip3/Nix (BNIP3L); and (iv) quality control by degradation of misfolded proteins or again portion of damaged mitochondria by the proteolytic system with chaperones and proteases^20^. It has been reported that mitochondrial biogenesis was decrease involved in muscle atrophy, which was promoted by PGC-1α and AMPKα^21, 22^. However, the process of MQC including mitochondrial fusion, fission, biogenesis and mitophagy in CKD muscle atrophy is still unclear.

TCM has been reported to be effective for the treatment of muscle atrophy^23–26^. However, there was little information available in literature about whether Chinese herbal medicine with anti-muscle atrophy effect could affect MQC process in CKD. JPYS decoction has been widely used in treating malnutrition with spleen and kidney qi deficiency syndrome in CKD for many years. However, further study of its detailed anti-malnutrition and reversing muscle atrophy mechanism is still needed. Here, we aimed to examine how dysregulation of MQC process induces muscle wasting and whether JPYS decoction inhibits muscle atrophy through modulating the MQC process effectively.

## Results

### Changes in renal function

At the end of study, CKD group displayed significantly higher serum creatinine (Scr) and blood urea nitrogen (BUN) levels compared with the sham group. Interestingly, JPYS decoction was found to reduce the levels of Scr and BUN. However, the level of serum albumin (ALB) did not differ significantly between all groups (Table 1).

**Table 1:** Renal function data (means ± SD).

Group	SCr(µmol/l)	BUN(mmol/l)	ALB(g/l)
Sham	61.51 ± 21.83	7.31 ± 2.02	89.10 ± 16.55
CKD	158.00 ± 45.11***	16.96 ± 2.77***	80.84 ± 12.21
JPYS	96.38 ± 29.39^###^	7.77 ± 2.04^###^	85.24 ± 8.19

***P < 0.001 between Sham and CKD groups; ^###^P < 0.001 between CKD and JPYS groups.

### JPYS decoction improves muscle atrophy

The bodyweight of CKD group was significantly lower than that of sham group at the beginning of the treatment; however, there were no differences in bodyweight between CKD and JPYS groups. Interestingly, JPYS group showed obvious improvement of bodyweight on the treatment of 5 and 6 weeks when compared with the CKD group (Fig. 1a). The increase in bodyweight from adding JPYS included an increase in weight of gastrocnemius (Gastroc) and tibialis anterior (TA) muscles in CKD group (Fig. 1b,c). The improved muscle mass in JPYS group was confirmed by an increase in average cross-sectional area of myofibers in TA muscles in CKD group (Fig. 1d,e).

**Figure 1:** Effect of JPYS decoction on body weight, muscle wet weight and muscle fibre cross-sectional area in 5/6 nephrectomised rats. (**a**) Body weight. (**b**,**c**) Weight of the gastrocnemius and tibialis anterior muscles was normalized by tibia length. (**d**) HE staining of the TA muscle. Scale bar = 100 μm. (**e**) Average fiber size of the HE-stained TA muscle. Results are presented as mean ± SD, n = 10 per group, a P < 0.05, b P < 0.001 between Sham and CKD groups, c P < 0.05 between CKD and JPYS groups; *P < 0.05, ***P < 0.001 between Sham and CKD groups. ^#^P < 0.05 between CKD and JPYS groups.

### JPYS decoction increases protein synthesis and suppresses protein degradation

The protein synthesis rate was lower in the CKD group than that of sham group, and JPYS decoction was found to increase the rate of protein synthesis (Fig. 2a). On the other hand, the protein degradation rate was higher in CKD group than in the sham group, which was completely inhibited by JPYS decoction (Fig. 2b).

**Figure 2:** Effect of JPYS decoction on muscle protein synthesis and protein degradation in 5/6 nephrectomised rats. (**a**) Protein synthesis was measured from the rate of incorporation of L-[U-^14^C] phenylalanine into isolated, incubated soleus muscles. (**b**) Protein degradation was measured as the rate of tyrosine released from isolated soleus muscles. Results are presented as mean ± SD, n = 6 per group, *P < 0.05 between Sham and CKD groups. ^#^P < 0.05 between CKD and JPYS groups.

### JPYS decoction inhibits ubiquitin-proteasome system and FoxO3a activation

Protein markers in muscle ubiquitin-proteasome system and FoxO3a are presented in Fig. 3a. CKD group displayed an increase in the expression of Atrogin-1 and MuRF-1, and these changes were abolished by JPYS decoction (Fig. 3b,c). Also, to confirm the relevance of the changes in muscle proteolysis seen in the CKD rats, we measured the activities of the 20 S proteasome. Both chymotrypsin- and trypsin-like activities was higher in CKD group than that of sham group, while were weakened with JPYS decoction (Fig. 3g,h). Additionally, the phosphorylated (p)-FoxO3a and p-FoxO3a/FoxO3a ratio were decreased in CKD group, while JPYS decoction trigger an increase as compared to the CKD group (Fig. 3d,f). As shown in Fig. 3e, basal protein content of FoxO3a was up-regulated in CKD group, and this was also prevented by JPYS decoction.

**Figure 3:** Effect of JPYS decoction on FoxO3a and ubiquitin-proteasome pathway in skeletal muscle of 5/6 nephrectomised rats. (**a**) Representative Western blot images of Atrogin-1, MuRF1, phosphorylated (p) form of FoxO3a and FoxO3a protein expression. (**b**) Quantification of Atrogin-1, (c) MuRF1 protein levels. (**d**) Quantification of p-FoxO3a, (**e**) FoxO3a protein levels and (**f**) FoxO3a/p-FoxO3a ratio. GAPDH was used as loading control. Data are expressed as Fold change vs. Sham and reported as means ± SD, n = 6 per group. (**g**) Chymotrypsin-like activity of the 20 S proteasome in gastrocnemius muscle was measured by using the fluorogenic substrate N-succinyl-Leu-Leu-Val-Tyr-7-amido-4-methylcoumarin. (**h**) Trypsin-like activity of the 20 S proteasome was measured by using the Boc-Leu-Arg-Arg-7-amido-4-methylcoumarin. Results are presented as mean ± SD, n = 6 per group, *P < 0.05, ***P < 0.001 between Sham and CKD groups. ^#^P < 0.05 between CKD and JPYS groups.

### JPYS decoction improves muscle mitochondrial content and aberrant muscle morphological features

Mitochondrial content was assessed using SDH staining of Gastroc muscles (Fig. 4a). The SDH activity, which represents mitochondrial amount, was markedly reduced in CKD group and JPYS decoction antagonized this response (Fig. 4b). On the other hand, SDH staining revealed that type I (slow oxidative) and IIa (fast oxidative glycolytic) muscle fibers, which are mitochondria-rich fibers, were significantly decreased, and type IIb (fast glycolytic) fibers were increased in CKD group. Quite interestingly, JPYS decoction displayed a shift in muscle fiber type in CKD group, characterized by a reduction in type IIb fibers and a significant increase in type I and IIa muscle fibers (Fig. 4c). Consistent with the decrease in SDH activity, the TEM morphologic also revealed major alterations at the sarcomeric level, with abnormalities consistent with fewer and smaller mitochondria (black arrows; Fig. 4e,f) and with markedly thinner Z-lines (white arrows; Fig. 4d) in CKD group. Similarly, the I-band, mainly constituted of thin actin filaments, appeared thinner or completely absent in CKD group (brackets; Fig. 4d). Importantly, these changes were prevented by JPYS decoction treatment.

**Figure 4:** Effect of JPYS decoction on skeletal muscle mitochondrial content and fiber type in 5/6 nephrectomised rats. (**a**) SDH staining was performed on 10 μm-thick sections from gastrocnemius muscles frozen in liquid nitrogen-cooled isopentane. (**b**) Quantification of SDH-stain intensity (expressed in A.U) and (**c**) number of type I (slow oxidative), and IIa (fast oxidative glycolytic) muscle fibers and type IIb (fast glycolytic) muscle fibers was assessed. Scale bar: 100 μm. Electron microscopy micrographs (magnification: 12,000x) of Gastroc muscles (**d**). Black arrows indicate mitochondria. Scale bar: 1 µm. Quantification of mitochondrial amount (number per field) (**e**) and size (average diameter, nm) (**f**) were performed. Results are presented as mean ± SD, n = 6 per group, *P < 0.05, **P < 0.01, ***P < 0.001 between Sham and CKD groups. ^#^P < 0.05, ^##^P < 0.01, ^###^P < 0.001 between CKD and JPYS groups.

### JPYS decoction increases mitochondrial biogenesis

Protein markers in muscle mitochondrial biogenesis are presented in Fig. 5a. The Cox IV protein can be used effectively as a mitochondrial loading control and represent mitochondrial content, which was consistent with the results of SDH activity (Fig. 5b). Additionally, mitochondrial biogenesis proteins NRF-1 and PGC-1α were also decreased in CKD group and these changes were reversed with JPYS decoction (Fig. 5c–e). However, the protein levels for the ATP5B and p-AMPKα/AMPKα ration were unchanged from all groups (Fig. 5d–f).

**Figure 5:** Effect of JPYS decoction on skeletal muscle mitochondrial biogenesis proteins in 5/6 nephrectomised rats. (**a**) Representative Western blot images of Cox IV, NRF-1, ATP5B, PGC-1α, phosphorylated (p) form of AMPKα and AMPKα protein expression. (**b**) Quantification of Cox IV, (**c**) NRF-1, (**d**) ATP5B, (**e**) PGC-1α protein levels and (**f**) p-AMPKα and AMPKα ratio. GAPDH was used as loading control. Data are expressed as Fold change vs. Sham and reported as means ± SD, n = 6 per group, *P < 0.05, **P < 0.05 between Sham and CKD groups. ^#^P < 0.05 between CKD and JPYS groups.

### JPYS decoction inhibits autophagy and mitophagy pathway

The autophagy and mitophagy-related proteins were detected by Western blotting (Fig. 6a). The level of Beclin-1 protein and LC3II/LC3I ration were up-regulated in CKD group and this was retarded by JPYS decoction (Fig. 6b,c). The contribution of the autophagy adaptor p62 has been found to be dispensable for mitophagy, which was incraeased in CKD group and attenuated by JPYS decoction (Fig. 6d). Interestingly, the levels of PINK1 and Parkin proteins were significantly increased in CKD group, and these changes were prevented by JPYS decoction (Fig. 6f,g). However, there were no differences in BNIP3L expression between all groups (Fig. 6e).

**Figure 6:** Effect of JPYS decoction on skeletal muscle autophagy/mitophagy pathway in 5/6 nephrectomised rats. (**a**) Representative Western blot images of LC3B, Beclin1, P62, BNIP3L, PINK1 and Parkin protein expression. Quantification of (**b**) LC3II/LC3I ration, (**c**) Beclin1, (**d**) P62, (**e**) BNIP3L, (**f**) PINK1 and (**g**) Parkin protein levels. GAPDH was used as loading control. Data are expressed as Fold change vs. Sham and reported as means ± SD, n = 6 per group, *P < 0.05, **P < 0.05 between Sham and CKD groups. ^#^P < 0.05 between CKD and JPYS groups.

### JPYS decoction decreases mitochondrial fission and increases mitochondrial fusion

The mitochondrial fusion and fission-related proteins were detected by Western blotting (Fig. 7a). The key fission proteins Fis-1 and Drp-1 levels were significantly higher in CKD group, while these changes were impeded by JPYS treatment (Fig. 7b,c). However, the key fusion proteins OPA-1 and Mfn-2 levels were decreased in CKD group, and this reduction was prevented by JPYS treatment (Fig. 7d,e).

**Figure 7:** Effect of JPYS decoction on skeletal muscle mitochondrial dynamics in 5/6 nephrectomised rats. (**a**) Representative Western blot images of Fis-1, Drp1, Opa1 and Mfn2 protein expression. Quantification of (**b**) Fis-1, (**c**) Drp1, (**d**) Opa1 and (**e**) Mfn2 protein levels. GAPDH was used as loading control. Data are expressed as Fold change vs. Sham and reported as means ± SD, n = 6 per group, *P < 0.05, ***P < 0.001 between Sham and CKD groups. ^#^P < 0.05, ^##^P < 0.01 between CKD and JPYS groups.

## Discussion

Many crude extracts and isolated active compounds from TCM have been identified and shown the excellent efficacy especially in anti-inflammation and metabolic disorder improvement for various types of kidney diseases^27–33^. Muscle atrophy is a serious complication of CKD patients, which is characterized by progressive loss of muscle proteins. This adverse outcome substantially reduces the quality of life and survival^16, 34^. The most important features of muscle atrophy are a significant reduction in body weight and loss of muscle mass, implying a CKD associated metabolic condition that specifically targets muscle. As a TCM, JPYS decoction has emerged as a potential therapeutic agent to treat muscle atrophy and increase muscle mass. To investigate the anti-muscle atrophy effect of JPYS decoction and its possible mechanism, in the present study, 5/6nephrectomy-induced CKD rats were performed, and results have shown that JPYS decoction considerably prevented body weight loss, muscle mass loss, muscle fiber size decrease, and muscle protein proteolysis, along with inhibition of UPS and FoxO3a. Moreover, JPYS decoction could increase mitochondrial content and biogenesis, restore the balance between fission and fusion, and block activation of autophagy and mitophagy.

Skeletal muscle mass depends upon a dynamic balance between protein synthesis and degradation. And the two processes are tightly interrelated^35^. The present results showed that JPYS decoction was able to increase protein synthesis and concomitantly inhibit breakdown of muscle in CKD rats. To investigate the underline mechanisms of delaying protein degradation by JPYS decoction, we examined the pathways of protein degradation. Increased Atrogin-1 and MuRF-1 promoted the ubiquitination and 26 S proteasome-mediated degradation of structural proteins, which increased muscle protein degradation and thus contributing to muscle wasting in our previous studies^36, 37^. Ubiquitinated proteins are rapidly degraded by the 20 S proteasome including chymotrypsin- and trypsin-like activities, that leading to Ub-conjugated proteins into small peptides^38^. In this study, our results showed that JPYS decoction prevented the elevated atrogin-1 and MuRF-1 proteins and chymotrypsin- and trypsin-like activities in CKD muscle. Previous studies identified that TCM (Zhimu-Huangbai Herb-Pair) treatment inhibited the Atrogin-1and MuRF1 expression in cancer-induced cachexia in mice muscle. These findings suggested that JPYS decoction could inhibit muscle protein degradation through inhibiting the activation of UPS in CKD rats.

FoxO3a can be phosphorylated by Akt at several sites, which functions as a scaffold within the cytoplasm, and are sequestered within the cytosol, rendering them unable to bind to the promoters of their target genes in the nucleus to regulate their transcription^39^. Previous study showed that the activation of FoxO3a in muscle leads to increased transcription of these atrogenes such as Atrogin-1 and MuRF1 and stimulates proteolysis to affect muscle atrophy^40^. Our result showed that JPYS decoction significantly increased the phosphorylation levels of FoxO3a, attenuated the level of total FoxO3a protein in the muscle of CKD rats. Previous study reported that TCM (Zhimu-Huangbai Herb-Pair) treatment reduced the expression of total FoxO3 protein in diabetic muscle^26^. It was reported that constitutively active FoxO3a induced atrogin-1 transcription and muscle atrophy, whereas inhibiting of FoxO3a activation blocked muscle atrophy *in vivo* and *in vitro* ^40^. Combining with the results we concluded that JPYS decoction could efficiently reduce protein degradation of skeletal muscle, possibly through inhibition of FoxO3a transcription factors.

The ability of skeletal muscle to adapt to cellular perturbations is highly dependent on mitochondrial biogenesis. It has recently been shown that muscle mitochondrial amount declines with CKD^41, 42^, which was consistent with our results, and the reduction was inhibited by JPYS decoction. The major steps of mitochondrial biogenesis process include signaling events leading to transcriptional regulation of nuclear genes, such as NRF1, mainly mediated by PGC-1α^43^. Our results showed that mitochondrial biogenesis proteins appeared to be down-regulated in CKD muscle as indicated by the lower PGC-1α and its target proteins NRF-1 content, which was inhibited by JPYS decoction. Overexpression of PGC-1α in skeletal muscle increases mitochondrial content and oxidative capacity through its modulation of a large group of genes involved in metabolism^44, 45^. Moreover, PGC-1a levels tend to be reduced in muscle wasting conditions^46, 47^ and muscle-specific overexpression of PGC-1a has been shown to attenuate this muscle loss^48^. Collectively, our data implied that it is possible that JPYS decoction promotes expression of PGC-1α/NRF1 and subsequent mitochondrial biogenesis in CKD muscle.

Autophagy/mitophagy is a highly conserved homeostatic mechanism that is used for the degradation and recycling, through the lysosomal machinery of bulk cytoplasm, long-lived proteins, mitochondria and organelles^49^. The selectivity of mitophagy is controlled by the proteins PINK1, Parkin and BNIP3L. PINK1 phosphorylates ubiquitin at Ser65 of ubiquitinated outer mitochondrial membrane (OMM) proteins and the ubiquitin-like domain of Parkin. Once phosphorylated, Parkin enhances the mitophagy signal by generating more ubiquitin chains on OMM proteins that can be further substrates for PINK1. BNIP3L is stabilized on the OMM, interacts with processed LC3II, which can promote sequestration of mitochondria within the autophagosome for degradation^9^. In our study, the results showed that the autophagic markers LC3II and p62, and mitophagic markers PINK1 and Parkin were significantly increased in CKD muscle, and this was retarded by JPYS decoction. Recent studies have demonstrated that autophagy, including mitophagy, is often stimulated in multiple models of muscle atrophy, such as denervation and CKD^37, 50^. Collectively, our results suggested that JPYS decoction improved muscle atrophy through inhibition of the autophagy and mitophagy pathway.

Mitochondria are reported to be highly dynamic organelles that undergo constant movement through fission and fusion^51^. Mitochondrial fusion is thought to allow the exchanging of their content including the mitochondrial DNA (mtDNA) and proteins, thus maintaining mitochondrial quality and mtDNA integrity, Mitochondrial fusion is thought to preventing accumulation of damaged and defective components through redistributing their content including the mitochondrial DNA (mtDNA), lipids, metabolites and proteins, whereas mitochondrial fission allows mitochondria for segregation of severely damaged and dysfunctional mitochondria by mitophagy^52^. In the present study, we demonstrated that the fusion protein Mfn-2 and OPA-1 were down-regulated in CKD muscle, and this change was prevented by JPYS decoction. Mfn2 and OPA-1 play an important role in maintaining mtDNA integrity, and their down-regulation could induce mitochondrial fission as well as mitochondrial fragmentation and mitophagy^53^. In accordance with a role in mitochondrial fusion, fission has been linked to the removal of severely damaged mitochondria through induction of mitophagy. In fact, our results showed that Fis-1 and Drp-1 expression were increased CKD muscle and this was prevented by JPYS decoction, which was consistent with our results^50, 54^. Therefore, the results of the present study indicate that JPYS decoction modulated mitochondrial dynamics of fusion and fission by increasing Mfn2 and OPA-1 expression, meanwhile decreasing Fis-1 and Drp-1 expression.

In conclusion, the present study show that a 6-week JPYS decoction treatment preserved the body weight, prevented muscle mass loss and muscle fiber size decrease, and muscle protein degradation, along with inhibition of FoxO3a and UPS in CKD rats. Furthermore, JPYS decoction attenuated the CKD-induced disturbances of MQC processes, by increasing mitochondrial biogenesis, restoring the balance between fission and fusion, and inhibiting autophagy-lysosome pathway (mitophagy). This finding suggests a promising strategy that improving the dysregulation of MQC processes might prevent and treat muscle atrophy in CKD.

## Materials and Methods

### Composition of JPYS decoction

Plant materials: Astragali Radix (Lot. 150621; roots of Astragalus membranaceus (Fisch.) Bge. var. mongholicus (Bge.) Hsiao), Atractylodis Macrocephalae Rhizoma (Lot. 141230; rhizomes of Atractylodes macrocephala Koidz.), Dioscoreae Rhizoma (Lot. 150615; rhizomes of Dioscorea opposite Thunb.), Cistanches Herba (Lot. 150621; herbs of Cistanche deserticola Y.C. Ma), Amomi Fructus Rotundus (Lot. 150617; fruits of Amomum kravanh Pierre ex Gagnep.), Salviae Miltiorrhizae Radix et Rhizoma (Lot. 150626; roots and rhizomes of Salvia miltiorrhiza Bge.), Rhei Radix et Rhizoma (Lot. 150104; roots and rhizomes of Rheum palmatum L.), and Glycyrrhizae Radix et Rhizoma Praeparata cum Melle (Lot. 150615; roots and rhizomes of Glycyrrhiza uralensis Fisch.) were purchase from Shenzhen Huahui Pharmaceutical Co., Ltd (Shenzhen, China). The plant materials were authenticated by Dr. Jianping Chen based on their morphological characteristics. The voucher specimens were kept at Pharmaceutical Department, Shenzhen Traditional Chinese Medicine Hospital with number 2010015Z, 2010024ZZ, 2010037Z, 2040056Z, 202086Z, 2010006Z, 2010040Z, and 2010008ZZ, respectively. Assurance of quality control for all the materials was validated according to the Chinese Pharmacopeia (China Pharmacopoeia Committee, 2015). Astragali Radix (30 g), Atractylodis Macrocephalae Rhizoma (10 g), Dioscoreae Rhizoma (30 g), Cistanches Herba (10 g), Amomi Fructus Rotundus (10 g), Salviae Miltiorrhizae Radix et Rhizoma (15 g), Rhei Radix et Rhizoma (10 g), and Glycyrrhizae Radix et Rhizoma Praeparata cum Melle (6 g) were weighed and extracted in boiling water (1.2 L) twice for 1 h. After centrigugation, the supernatant was dried under reduced pressure to powder, and it was stored at −80 °C. Before the treatment, the powder was re-dissolved with Milli-Q water and vortexed at room temperature to obtain JPYS extract.

Before the treatment of extract onto animals, JPYS extract was chemically standardized. An HPLC fingerprint at 260 nm was developed for the JPYSF extract (Fig. 8): An individual reference standard was employed to confirm numerous chemical components should be identified from the extract by HPLC analysis, such as sodium danshensu, echinacoside, acteoside, calycosin 7-O-b-glucoside, salvianolic acid B, formononetin and rhein. Besides, the minimal requirement for the amounts of echinacoside, salvianolic acid B and rhein should be no less than 1.2 mg/g, 5.7 mg/g and 0.2 mg/g of the dried extract. The yield of the extraction was less than 32.59 ± 1.1% (w/w, Mean ± SD, *n = *3). The extract being used here reached the aforesaid requirements.

**Figure 8:** The main components of JPYS decoction extract were determined by HPLC. (**a**) Chemical structure of the main active ingredients of JPYS decoction. The denotation peaks 1–7 were sodium danshensu (1), echinacoside (2), acteoside (3), Calycosin-7-O-β-D-glucopyranosid (4), salvianolic acid B (5), formononetin (6) and rhein (7). (**b**) HPLC fingerprint profile of JPYS decoction extract at 260 nm.

### Experimental animals

The experimental and feeding protocols were in accordance with National Health guidelines and were approved by the Guangzhou University of Chinese Medicine Institutional Animal Care and Use Committee. Male Sprague–Dawley rats were purchased from Guangdong Medical Laboratory Animal Center (GDMLAC, China), Permission No. SCXK (YUE) 2013-0002 weighing 190–220 g. The animals were under controlled room temperature (20 ± 1 °C) and with humidity with 12/12-hour light-dark cycle, and had access to water and food ad libitum. CKD was induced by a two-step 5/6 nephrectomy as our described previously^36^. Briefly, the first renal surgery involved electrocautery of the left kidney except for a 2-mm area around the hilum. A second renal surgery was performed one week later by double ligation of the renal hilum with silk suture and surgical excision of the right kidney. Sham surgery consisted of anesthetic, flank incision exposing the kidney and closure of the abdominal wall.

### Administration of drugs

At 16 weeks after the operation, the levels of Scr of the 5/6 nephrectomy group was significantly higher than those of sham group (p < 0.05). Then, the 5/6 nephrectomy group was randomly divided into two groups: CKD group (5/6 NX, n = 10): CKD rats were treated with distilled water and JPYS group (5/6 NX + JPYS decoction, n = 10): CKD rats that were orally administrated a dose of 10.89 mg/kg of JPYS decoction daily. The sham-operated rats were also treated with distilled water. The drugs were administered for 6 weeks. All rats used in this study received humane cares.

### Biochemical parameters

After 6 weeks treatment, the rats were sacrificed by sodium pentobarbital and blood samples were collected immediately. Serum biochemical indexes Scr, BUN and ALB were detected using a Roche automatic biochemical analyzer.

### Morphological studies (HE, SDH staining)

The transverse paraffinized muscle sections (6 mm) were stained with hematoxylin and eosin (HE) in line with standards. Muscle fiber cross-sectional area (CSA) was then measured in the way as our previously reported^37^. Fiber cross-sectional area was measured for approximately 100 adjacent muscle fibers in each section for each mouse using Image J 1.32 j software (NIH, Bethesda, MD, USA).

The frozen sections of the TA muscle was stained with succinate dehydrogenase (SDH, complex II of the respiratory chain) for measurements of SDH activity and classification of fiber type into I (slow oxidative), IIa (fast oxidative glycolytic) or IIb (fast glycolytic) in accordance with a previously described protocol^41^. Briefly, sections were first allowed to reach room temperature and were rehydrated with PBS (pH 7.4). Sections were then incubated in a solution containing nitroblue tetrazolium (1.5 mM), sodium succinate (130 mM), phenazine methosulphate (0.2 mM) and Sodium azide (0.1 mM) for 60 min. Cross-sections were then washed 3 times in PBS, dehydrated in 75% (30 s), 90% (30 s) and 100% (10 min) ethanol and cover-slipped with a mixture of 50% (v/v) glycerin and 2.5% (w/v) triethylene diamine in 0.01 M PBS. Images of muscle were captured using a microscope (Nikon Eclipse Ti-SR, Japan) and were digitized as gray-level images on a computer assisted NIS-Elements imaging software Version 4.10 (Eclipse Ti-SR, Nikon Corporation, Tokyo, Japan). A gray level value of zero was equivalent to 100% transmission of light (%T), and that of 255 was equivalent to 0%T. The optical density value of all the muscle fibers was determined based on the gray-level images (Scion image, Scion, Frederick, MD) and classified into three groups, I (%T: 100–80%), IIa (%T: 60–40%) and IIb (%T: 20–0%).

### Ultrastructural analysis (Transmission Electron Microscopy, TEM)

Detailed procedures of TEM for muscle were as our previously reported^55^. Briefly, sections of TA muscle 1 mm^3^ in volume were fixed in 2.5% glutaraldehyde followed by postfixation in 1% osmic acid for the assays of electromicroscopy. Image J software was used to analyze images collected by EM (JEM-1400, JEOL Ltd.,Tokyo, Japan) under x12,000 magnification. Mitochondrial content was determined by quantifying the number and the size (minimum diameter) of each mitochondria per field. A total of 20 fields per condition were analyzed by taking advantage of the Image J software^56^.

### Protein synthesis and protein degradation

Protein synthesis and protein degradation were measured *in vitro* using the incorporation of 14-C phenylalanine (phe) and tyrosine release as previously described^57–59^.

### Measurement of proteasome activities

The chrymotrypsin- and the trypsin-like activity of the 20 S proteasome were measured *in vitro* in the gastrocnemius muscle as our previously described^36^.

### Western blotting

Snap-frozen quadriceps muscle tissues were homogenized in lysis buffer as our previously reported^36^. Cytosolic proteins were separated on a 10% SDS-PAGE gel and then transferred to a PVDF membrane (Bio-Rad Laboratories, Hercules, CA, U.S.). The membrane’s nonspecific binding sites were blocked at room temperature for 1 h with 5% non-fat powdered milk in Tris buffered saline with tween (TBST) and then incubated overnight at 4 °C with primary antibodies. After washed with TBST, the membranes were incubated with secondary antibodies for 1 h at room temperature with shaking. After washing, protein bands were detected and analyzed using a ChemiDoc™ MP Imaging System (Bio-Rad Laboratories, CA, U. S.). Results were expressed as the integrated optical density relative to GAPDH. p-AMPKα (1:1000, #2535), p-FoxO3a (1:1000, #13129), SQSTM1/p62 (1:1000, #5114), Mitofusin-2 (1:1000, #9482), FoxO3a (1:1000, #2497), DRP1 (1:1000, #8570), Cox IV (1:1000, #4844), BNIP3L/Nix (1:1000, #12396) Beclin-1(1:1000, #3495 T) and AMPKα (1:1000, #5831) antibody were from Cell Signaling Technologies (Danvers, MA, U.S.). LC3 I/II (1:1000, ab58610), Parkin (1:1000, ab77924) and PINK1 (1:1000, ab23707) antibody were from Abcam (Cambridge, U.K.). ATP5B (1:1000, ARP48185_T100) antibody was from Aviva Systems Biology (San Diego, CA, U.S.). MuRF1 (1:1000, GTX110475) antibody was from Gene Tex (San Antonio, TX, U.S.). Fis1 (1:100, sc-98900) and NRF-1 (1:100, sc-33771) antibody were from Santa Cruz Biotechnology (CA, U.S.). OPA1 (1:1000, 612606) was from BD Biosciences (San Jose, CA, U.S.). Atrogin-1 (1:1000, AP2041) was from ECM Biosciences (Versailles, KY, U.S.). PGC-1α (1:2000, NBP1-04676) was from Novus Biological (Colorado, U.S.). GAPDH (1:1000, 60004-1-Ig) was from Proteintech (Chicago, IL, U.S.).

### Statistical analysis

Data were analyzed with SPSS 16.0 (SPSS Inc., Chicago, IL, USA). Results are shown as mean ± SD. Normally distributed data were analyzed by one way ANOVA followed by Least-significant Difference (LSD) test, while data without normal distribution were analyzed using Games-Howell test. Differences were considered statistically significant for P < 0.05.
